# The past, present and future of protein-based materials

**DOI:** 10.1098/rsob.180113

**Published:** 2018-10-31

**Authors:** Nadia C. Abascal, Lynne Regan

**Affiliations:** 1 Department of Molecular Biophysics and Biochemistry, Yale University, New Haven, CT, USA; 2 Department of Interdisciplinary Science, Centre for Synthetic and Systems Biology, Institute for Quantitative Biology, Biochemistry and Biotechnology, School of Biological Sciences, University of Edinburgh, Edinburgh, UK

**Keywords:** protein-based materials, recombinant proteins, biomaterials, drug delivery

## Abstract

Protein-based materials are finding new uses and applications after millennia of impacting the daily life of humans. Some of the earliest uses of protein-based materials are still evident in silk and wool textiles and leather goods. Today, even as silks, wools and leathers are still be used in traditional ways, these proteins are now seen as promising materials for biomaterials, vehicles of drug delivery and components of high-tech fabrics. With the advent of biosynthetic methods and streamlined means of protein purification, protein-based materials—recombinant and otherwise—are being used in a host of applications at the cutting edge of medicine, electronics, materials science and even fashion. This commentary aims to discuss a handful of these applications while taking a critical look at where protein-based materials may be used in the future.

## 1. Introduction

Protein-based materials have had a place in society for millennia. Silk, wool and leather are particularly notable examples, obtained by the age-old practices of cultivating silkworms for silk production, raising sheep for wool production, and using a hunt's catch to obtain leather hides. These materials have exceptional physical properties, with the huge advantage that they are intrinsically biodegradable and are ultimately returned to the biomass of the earth. There is therefore currently much interest in both manufacturing new protein-based materials and obtaining familiar materials in different ways.

Silk has been used for centuries to create fine textiles not only due to its aesthetic quality and rarity, but also—and perhaps most importantly—its strength. Silkworms, the caterpillar larvae of *B. mori* moths, are still cultivated for silk production using culture methods that have changed little over several thousand years. While effective, the methods are time-intensive and not readily scalable. A key step in the production of silk is to harvest the cocoons (by boiling or piercing them to kill the larvae) at the optimal time in their development, so that the silk can be unwound as essentially one single long thread [1].

Although the processes to make leather are typically performed on a much larger scale, tanning is both time-intensive and noxious. Many of the chemicals and biological that are needed to strip leather away from materials, such as hair and extraneous fibres, are malodorous, harsh and toxic [2]. Leather production has always been driven by meat production, but a synthetic process could circumvent that tandem supply-and-demand relationship. Those who like the look and feel of leather but are opposed to its method of production have driven the development of a purely synthetic alternative. Additionally, creating new materials from the component proteins of materials like silk, wool and leather holds promise in the area of textiles and beyond.

Until recently, the concept of using natural fibres—or synthetic materials derived from them—as ‘smart materials’ was still an underdeveloped area of research. Today, the literature is exploding with new designs for protein-based materials for a variety of applications. The ease with which researchers can programme the expression of any protein has made using proteins in a wide array of biomaterial applications appealing [3]. In addition to being accessible and part of a circular economy of source materials, protein-based materials are biocompatible and biodegradable—qualities that are highly attractive [4]. Furthermore, because many structural proteins are polymeric materials composed of discrete repeats of amino acid sequences, they are highly modular, which facilitates easy manipulation [5]. A specific amino acid sequence that is found to impart appealing characteristics can often be fused with another protein, thus combining the attractive qualities of both; for example, combining a sequence that gives a protein its strength with another that gives it its elasticity can give rise to a strong, yet stretchy, material. The intrinsic strength and elasticity of natural proteins such as silk, elastin, resilin, collagen and keratin have put these proteins at the centre of such research [3]. Additionally, composite materials that are silk-, elastin-, resilin-, collagen-, keratin-like or some combination thereof, or which incorporate inorganic components, is also proving to be promising in many biomaterial applications [3].

Herein, we take a non-exhaustive look at the cutting edge of the research and development of protein-based materials. Both natural fibres and synthetically produced materials will be considered, with regard to a variety of applications, and the advantages and limitations of their use.

## 2. Material composition

The structural compositions of the most common proteins used in materials (i.e. silk, elastin, resilin, collagen and keratin) all have hallmark features that underlie their exceptional mechanical strength and elasticity (figure 1). The unique properties of these proteins are inherently linked to their composition, typically multiple tandem repeats of short amino acid sequences. Depending on how these amino acids are linked, a protein will be imbued with specific qualities, atypical of common globular proteins.

**Figure 1.** All of the materials presented here have natural sources and conserved, repeated amino acids in their primary structures.

### 2.1. Silk composition

Silk, comprised two distinct components: the core protein fibroin and its glue-like coating sericin, which is removed before the fibre is processed into usable materials. Some researchers are independently investigating sericin itself for potential uses as a material, [6] but our focus is on fibroin-based materials [7].

The key components of fibroin, which underlie its mechanical properties, are the tightly packed, antiparallel β-sheets, sometimes referred to as crystallites, formed by the glycine and alanine-rich repeat regions of the protein (figure 1) [8].

### 2.2. Elastin composition

Elastin is a major mammalian structural protein that is present in blood vessels, lung epithelium, skin and other tissues [9]. On a structural level, elastin is made up of tandem tetra-, penta- and hexa-repeats of discrete peptide sequences composed of predominantly hydrophobic residues, such as valine, alanine, glycine and proline. These sequences are interspersed with more hydrophilic domains that are rich in lysine and alanine repeats [10]. Models of elastin have suggested that stretching decreases entropy (i.e. expels water molecules from the structure) such that there would be an entropic driving force for elastin's hallmark elasticity [11,12].

### 2.3. Resilin composition

Resilin is a pliable and extendable structural protein found in insects. It is named for its resilience to repeated rounds of stretching and relaxation. Resilin's ability to store mechanical energy gives insects their ability to efficiently jump and fly [13]. Resilin has three domains, which consist of an N-terminal domain with eighteen 11-amino acid repeats (exon I), a middle chitin-binding domain (exon II) and a C-terminal domain with eleven 13-amino acid repeats (exon III). The N-and C-terminal repeat containing domains seem to be key to the protein's unique properties. Exon I is the elastic, very resilient, ‘soft’ domain, whereas the C-terminal domain is ‘hard’ and significantly less resilient. Experiments where the sequence of the repeats is changed there have identified a threshold of glycine and proline content above which the repeat structures are elastic. Both the N- and C-terminal domains are predicted to be disordered, with the N-terminal domain additionally being predicted to have some propensity for β-turn structure [14].

Upon a thermal stimulus or mechanical stress, exon III can transform to a more ordered β-turn structure. The associated energy is converted into kinetic energy to be used in insect jumping or flying. Following the use of this kinetic energy, exon III cools and relaxes, returning to its original conformation [14]. Resilin's primary structure is conserved to some degree across different insects, in that YGAP repeats are common in the N-terminal domain [15]. However, the exact sequence of the resilin varies from source to source (i.e. mosquito resilin varies from fruit fly resilin), although one of the most commonly used repeat sequences for recombinant resilin is that from *A. gambiae*, AQTPSSQYGAP [16].

### 2.4. Collagen composition

Like resilin, collagen is a highly conserved structural protein. It is the most abundant structural protein in mammalian tissues. The fundamental structure is three α-helical chains, which associate as either homo- or hetero-trimers [17]. These trimers then assemble into more complex supramolecular structures, including fibrils, beaded filaments, anchoring fibrils, networks and hexagonal networks [17]. The primary structure of collagen is dominated by glycine-X-Y repeats, where X is generally hydroxyproline and Y is proline [18]. The presence of hydroxyproline in collagen is thought to contribute to its thermostability; mutations that delete hydroxyproline from various points in the collagen sequence significantly decrease its thermal denaturation temperature [19].

### 2.5. Keratin composition

Keratin is another noteworthy protein in this class. It is a structural protein found in scales and claws of reptiles, beaks and feathers of birds (β-keratin), and hair and wool of mammals (α-keratin) [20]. Although both α- and β-keratin have in common that they are rich in the amino acid cysteine, and have fairly large numbers of disulfide cross-links, they are structurally quite different. α-keratin is a helical protein, which assembles into coiled coils and ultimately helical filaments. By contrast, β-keratin forms beta sheets, which also assemble into higher-order filaments. Both α- and β-keratin are typically embedded in an amorphous keratin matrix in their functional form. β-keratin can also be found in an amorphous form, and involved in other functions, including as the basis for structural colour in certain bird feathers.

Keratin's insolubility and ubiquity in agricultural waste products, such as chicken feathers and unsuitable wool, make it particularly attractive in biomaterial applications [20]. The presence of cell adhesion sequences arginine-glycine-aspartic acid (RGD) and leucine-aspartic acid-valine (LDV) in the natural sequence of keratin also add to its potential to be used as a matrix for cell growth [20]. The individual structural qualities of keratin, silk, elastin, resilin and collagen, as well as these materials' common characteristics of biocompatibility and biodegradability, all contribute to their presence at the forefront of biomaterials research.

## 3. Applications

Protein-based materials hold special promise in that they can be tuned and altered in their chemical composition as well as their morphology. The numerous ways in which the raw protein of these materials is processed allows researchers to manufacture a form of the protein that is best suited for a particular application. For example, protein can be processed such that its malleability and softness simulate conditions that encourage cell differentiation [21], thus adding another level to these materials’ biocompatibility and the breadth of their application.

Silks have been at the forefront of this type of research. One type of the many silks produced by spiders, dragline silk, is even stronger than the traditional silkworm-derived silk. Producing dragline silk from spiders is a much more daunting undertaking than producing traditional silk from silkworm. Dragline silk must be produced from individual spiders, which are difficult if not impossible to rear in captivity, and therefore the yields would be minuscule.

Consequently, there is great interest in developing methods to make both traditional silk and dragline silk recombinantly, with the potential for increased yields and a more consistent product. Although it has proven relatively easy to express recombinant fibroin (the key protein of silk), developing methods to generate fibres from these monomers is difficult. A variety of strategies are being pursued, including various procedures for processing and expression [22].

The gland responsible for making dragline silk in spiders is made up of a tail-like region and a wider sac [23]. The tail-like region secretes the so-called ‘spinning dope’, which is an aqueous solution of protein to make the silk fibre [23]. The sac acts as a repository and funnels the solution to a complex duct that ends in a valve [23]. While the duct's shearing force aids in condensing the protein into a solid material, a pH gradient (from 7.6 to less than 5.7) over the gland induces a conformational change in the fibroin, such that fibre formation is promoted [24]. Recapitulating such a mechanism to convert recombinant silk fibroin proteins into silk fibres, in a scalable fashion, is a major roadblock to producing large amounts of recombinant silk fabric. Bolt Threads has developed a proprietary method for producing dragline silk and has forged a contract with fashion designer Stella McCartney for a dragline silk clothing line (figure 2), with one dragline silk dress reported to date [1].

**Figure 2.** A dress designed by Stella McCartney using synthetic dragline silk. (Image via Bolt Threads.)

Various processes are being developed to use recombinant silk fibroin (most typically expressed in *E. coli*) in different applications, in addition to preparing threads for clothing (figure 3) [22]. Following lyophilization of purified fibroin, the protein can be treated and cast in multiple morphologies that are appropriate for specific applications. The fibroin can be electrospun into nanofibres, self-assembled or wet-spun into microfibres, self-assembled into hydrogels, solvent cast into mesoporous foams, desolvated to form particles, emulsified into capsules or cast into films [22]. These silk-based materials have been made into biodegradable screws or plates, via a solvent-based process, used in repairing bone fractures [25]. Dragline spider silk has also been used to make artificial skin [26]. Porous scaffolds, hydrogels, films and electrospun fibres have been used to encourage tissue growth during subcutaneous implantation, for example, in wound healing and tissue engineering endeavours [27,28]. The advantage of creating hydrogels from proteins is that function can be readily introduced into the structural matrix. For example, the RGD sequence can be introduced onto the protein to encourage cell attachment to the gel [28].

**Figure 3.** The forms synthetic silk-based and other protein-based materials can take through various treatments. (Image adapted with permission from Advanced Materials.)

Other proteins have also been investigated for their potential application in tissue engineering. Elastin and elastin-based materials can also be made into biocompatible electrospun fibres and hydrogels [3,29,30]. Additionally, elastin protein and elastin-like peptides are hydrophilic and cell-interactive via a positively charged GRKRK C-terminal domain, used in integrin binding [31]. Additionally, tweaking elastin's composite repeats with a variable residue allows for tuneable properties in elastin-like peptides [32].

Resilin and resilin-based materials have been made into hydrogels for potential use in tissue engineering [33]. A key feature of resilin structure is the presence of unusual tyrosine–tyrosine cross-links. These can be introduced into recombinant resilin materials using chemical oxidation, or the enzyme transglutamase. Using such cross-linking strategies, hydrogels, which mimic the elastic properties of the subendothelial layer of the vascular system, have been created from recombinant resilin, thereby providing a promising material for vascular tissue regeneration and long-term cell attachment [34].

Finally, collagen and collagen-based materials have found use in multiple applications in this realm including, quite successfully, in corneal implants [35]. Collagen has been used for tissue grafts and made into a porous gel that promotes tissue regrowth [36]. Recombinant collagen (expressed in yeast, or in plants) is an attractive alternative to collagen harvested from animals, and has few contaminants [37–39].

Furthermore, Modern Meadows has developed a method by which collagen protein produced by yeast cells can be purified and processed into leather sheets (figure 4) [2]. Their exact procedure is proprietary, but the company can produce a product that is no longer limited by the size and shape of an animal, nor by the supply of leather as a meat by product [2].

**Figure 4.** Synthetic leather produced by the company Modern Meadows. (Photo from http://www.modernmeadow.com/our-technology.)

In addition to these diverse applications, protein-based materials have also been used in drug delivery. Silk-based materials have been made into nanoparticles for this purpose and been expressed fused to various peptides to tune modes of delivery [3]. By expressing silk fibroin protein fused to a peptide that is negatively charged at physiological pH, drug delivery can be made pH dependent. The drug encapsulation efficiency of a positively charged drug is high at physiological pH, whereas in the low pH environment of a tumour, binding is weakened and the drug cargo is released [40]. Recombinant silk containing poly(l-lysine) domains has also been engineered to contain tumour cell-binding peptides so that DNA can be delivered in a target-specific fashion [40]. Elastin and elastin-based materials can be made into stimuli-responsive polymers by manipulation of amino acids added to elastin's modular repeat sequence, or by altering the repeat sequence itself [41]. Tracking how the properties change as a result of these modifications provides a deeper understanding of how the physical properties of the material are determined by the amino acid sequence [41–43].

Aside from tissue engineering and drug delivery, protein-based materials have shown promise as conductive and antimicrobial materials and packaging. Synthetic materials, comprised tandem repeats of amino acids, exhibit sought-after traits for applications in energy and electronic technologies [44]. For example, the tandem repeat sequences, motifs of alternating A, V, S, T, H-rich and G, L, Y-rich segments, derived from squid ring teeth proteins (a soft yet sturdy protein present in the suction cups squids' tentacles) which have been reported to exhibit the highest bulk proton conductivity of any biomaterial tested [44].

Keratin, or wool, can be easily functionalized via chlorination to produce a halamine-charged material [20]. In the form of textiles, films or nanofibres, halamine-charged keratin is anti-bacterial [20]. Furthermore, these materials maintain their potency even after repeated washing. Halamine-charged keratin could have an important role in the manufacturing of materials for a multitude of purposes [20].

Protein-based materials also provide an opportunity to re-purpose ‘protein-rich waste products’ in new applications. Many foods benefit from being ‘coated’ to maintain hydration and to prevent oxygen entry, because both these processes are associated with diminution of the quality of the product. Plastic-based wraps have been widely used, but as non-biodegradable products, after which they accumulate as waste. There is therefore significant interest in making coatings with suitable tensile strength and elasticity from protein sources that would otherwise be discarded. Such protein-based coatings, in addition to reducing spoilage, would ideally have no taste, and could therefore either be eaten along with the product they coat, or removed and biodegraded and returned to the earth. Two sources of excess proteinaceous material that would otherwise go to waste are casein in excess milk from the dairy industry, and keratin, in waste feathers from the poultry industry, both of which have the potential to be appropriated for use as food coatings and other applications. In these examples, these proteins are acquired from their original sources, but used in different formulations, to manufacture new materials [45,46].

Another aspect of protein-based materials, which is beginning to be explored, is the idea of combining more than one protein, to obtain a material that exhibits the desirable characteristics of both. One particularly noteworthy example is the silk-elastin-like peptides (SELPs), which have been electrospun and used to create biocompatible fibrous scaffolds with applications in tissue engineering [47,48], and also hydrogels and nanoparticles for drug delivery [49–51].

## 4. Perspectives and conclusion

The use of protein-based materials is becoming more prevalent across a wide range of fields and applications. The examples discussed above mainly concerned fibrous proteins; however, the potential to use globular proteins, with unusual physical properties, to create novel materials is also beginning to be exploited. BslA, a bacterial hydrophobin that self-assembles at hydrophobic/hydrophilic interfaces to form robust monolayers is one example. It has been shown to stabilize emulsion droplets, allowing the potential for drug delivery [52,53] and may even be used to coat ice cream to slow its melting [52,53]. More recently, protein-engineering strategies have been developed to functionalize BslA after it has assembled into a monolayer [54,55], allowing researchers to further extend the potential of BslA-based coatings to a wider range of applications, including sensing.

Protein-based materials offer myriad opportunities to tailor the macroscopic properties of a material by changing either the sequences of the proteins from which they are made, or the means by which they are processed. The scope of potential applications for such materials, some of which have been discussed in this review, is enormous. In addition, their intrinsic biodegradability and their role in a circular economy, turning products that would otherwise go to waste into useful new materials, are of inestimable importance. The dawn of self-cleaning fabrics that include lipase-doped protein-based fibres or wearable sensors that could alert a wearer of an impending medical emergency is closer to reality than it is to science fiction. Protein-based materials are advancing quickly to soon become the prominent options for problems of biomedical engineering, materials science, waste management and beyond.

## 5. Definitions

Many of the terms associated with biomaterials are quite loosely defined, with broad interpretations, while others are more precisely defined. It is therefore important to specify the meaning of a few commonly used terms in the field. Some of these terms appear in this commentary.

*Biocompatible.* A biocompatible material can interact with living cells or a living organism without eliciting a negative response. The definition of ‘a negative response’ is rather vague and tends to be application specific. Often, this term is used to describe materials that are used as scaffolds on which to grow cells and tissue, or in controlled drug release applications.

*Biodegradable*. A biodegradable material can be broken down by natural or biological processes. We use the term to imply that such degradation will occur ‘over a reasonable time scale’ and in a range of conditions. The term itself does not imply a particular time scale or efficiency of degradation in a given condition.

*Circular economy.* In a circular economy, materials are reused and recycled. For example, an otherwise waste product from one process is not discarded but used as feedstock for another process. It is perceived as a more sustainable alternative to the traditional linear economy (make, use and discard).

*Elastic modulus.* A material's resistance to being deformed elastically (i.e. reversibly) when subjected to a stress. The less elastic (i.e. more stiff) a material, the higher its elastic modulus.

*Electrospinning.* A way of producing very thin fibres, where charged threads of a polymer (or protein) solution are pulled towards an oppositely charged plate. Typically used on a small scale, but a handful of companies globally offer scaled-up facilities.

*Mesoporous.* The material has many intermediately sized pores (between 2 and 50 nm in diameter) [56].

*Self-cleaning*. A material that can react with a contaminant to render it benign. Often this means incorporating an enzyme into the material; for example, organophosphate degrading enzymes incorporated into filters to remove pesticides from water, or in protective clothing to counter nerve agent attacks.

*Self-healing.* A self-healing material will automatically repair any damage it incurs, without additional intervention. Many protein-based materials have an ability to continually repair themselves by spontaneously forming new bonds following a bond break. This phenomenon is often observed in protein-based hydrogels.

*Strain healing*. In repeated cycles of strain and relaxation, the material becomes stronger.The first cycle of stretching actually helps remove some imperfections, and upon relaxation the material is now improved.

*Tensile strength*. The maximum amount of stress a material can withstand before it breaks.

*Yield strength*. The point at which behaviour under stress is no longer elastic.

## Data accessibility

This commentary has no additional data.
